The article "Development of Deep Learning Technique of Features for the Analysis of Clinical Images Integrated with CANN" was retracted in 2024. Reasons: signs of a paper mill; suspected computer-generated content; unreliable results or conclusions; concerns about the data.

# Development of Deep Learning Technique of Features for the Analysis of Clinical Images Integrated with CANN

**DOI:** 10.1155/2022/2742274

**Published:** 2022-10-14

**Authors:** Prabakaran Kasinathan, R. Prabha, R. S. Sabeenian, K. Baskar, A. Ramkumar, Samson Alemayehu

**Affiliations:** ^1^Department of Computer Science and Engineering, School of Computing, Vel Tech Rangarajan Dr. Sagunthala R&D Institute of Science and Technology, Chennai, 600062 Tamil Nadu, India; ^2^Department of Electronics and Communication Engineering, Sri Sai Ram Institute of Technology, Chennai, 600044 Tamil Nadu, India; ^3^Department of Electronics and Communication Engineering, Sona College of Technology, Salem, 636005 Tamil Nadu, India; ^4^Department of Artificial Intelligence and Data Science, Kongunadu College of Engineering and Technology, Trichy, 621215 Tamil Nadu, India; ^5^Department of Electrical and Electronics Engineering, Kalasalingam Academy of Research and Education, Krishnankoil, Tamil Nadu, India; ^6^Department of Electrical and Computer Engineering, Faculty of Electrical and Biomedical Engineering, Institute of Technology, Hawassa University, Ethiopia

## Abstract

Computer tomography is an extensively used method for the detection of the disease in the subjects. Basically, computer-aided tomography depending on the artificial intelligence reveals its significance in smart health care monitoring system. Owing to its security and the private issue, analyzing the computed tomography dataset has become a tedious process. This study puts forward the convolutional autoencrypted deep learning neural network to assist unsupervised learning technique. By carrying out various experiments, our proposed method produces better results comparative to other traditional methods, which efficaciously solves the issues related to the artificial image description. Hence, the convolutional autoencoder is widely used in measuring the lumps in the bronchi. With the unsupervised machine learning, the extracted features are used for various applications.

## 1. Introduction

Computed tomography is a widely used method in recent years, in which clinician early examines the nature of the disease in a very systematic manner and the cause of the disease is also detected priorly. For each and every subject, there may be several images taken for examination due to this complexity and proper validation is not possible; thus, to solve this, smart medical management plays a vital role [1]. Primarily, detection of the lumps in the bronchi is of main task; hence, this helps in detecting the early stage of the tumor in the bronchi through the enormous quantity of the pneumatic computed tomography images. Thus, the examination of the images is done in several ways: (i) to define the ROI (region of interest), (ii) image segmentation, and (iii) manual feature extraction and finally classification [2]. In order to analyze the lump, the extraction of the features is performed. Considering the size, shape, and edges of the lump, the disease is classified. The systematic approach does not provide better results [3]. Medical expertise may produce a defective result in examining the disease. Thus, the feature extraction process helps in the analyses of the lump in the bronchi. Thus, convolution neural network plays a significant role in the determining the lump in the bronchi better than that of the manual feature extraction process. Hence, the numerous datasets are needed for this feature extraction process [4].

To overcome these challenges, an effective deep learning framework depending on convolutional autoencrypted neural network (CANN) was used for categorizing the lump in the bronchi [5]. The initial stage required for examining the lump in the bronchi uses the normal image, and then from the input image, the features are represented. In order to classify the lump in the bronchi, the computed tomography images are required and the spotted images are extracted. Each respective spot contains the particular set of results. The result proves that the suggested method is much effective in the feature extraction process [6]. The main essential of using convolutional autoencoder neural network rather than using CNN is to acquire the low-dimensional noiseless image representation and acquisition for the purpose of extracting its features and classification and hence would yield higher accuracy results. It also aids the added advantage of a unique case of an unsupervised learning model for reproducing the best noiseless input image with its adequate feature attribute values.

The illustration of the system defining the lack of unlabeled feature samples has been depicted in Figure 1. In addition to that, the illustration over the schematic block functional representation of CANN for medical image analysis has been depicted in Figure 2. From the actual computed tomography images, the spotted parts are thoughtlessly selected for the examination of the lumps in the bronchi. Thus, the labelling of the image and the region of the interest are calculated efficiently by the clinician [7]. Hence, there exists a lump in the respiratory track; thus, to solve this issue, the learning approach is implemented. In order to eliminate the huge amount of data obtained from manual feature extraction process, our proposed method uses CANN to avoid such issues; they are capable of effectively detecting the inadequacy in the training data. Through the original image, the feature extraction process is performed. This kind of extinguished method does not require segmentation process to detect the spot; these unsupervised data are used in other various applications [8]. Performance realizations over the various classifications as shown in Table 1.

## 2. Related Literature Survey

So as to obtain the extracted feature, the selection of features has to be done. Deep learning is an emerging work performed in the recent years. Comparative to the traditional method, the data-driven feature learning approach produces better results [9, 10]. With the help of the deep learning technique, the feature extraction process is carried from the original image datasets, and the intricate features are extracted by the reoccurring layers. Essentially, the representation learning is categorized into two types; one is unsupervised learning and supervised learning [11]. For the prediction purpose, the data are transmitted from the initial stage to the top most layer. The back propagation is the technique used for evaluating the cost function linking the predicted and the target value [12, 13]. CNN is basically used in speech identification, image examination, and text exploration. In the image examination, the CNN plays a vital role in face identifying, segmentation of the cell, identifying the breast images, and identifying the injury in the brain. Whereas in unsupervised learning to predict the features of the images, the unlabeled features are used and the fewer amount of supervised data are used for attenuating the parameters [14]. In this study, a convolutional autoencrypted learning algorithm is proposed to determine the features of the computed tomography bronchi images and to categorize the spot in the respiratory track. In our proposed study, the unsupervised autoencrypted feature and CNN were combined to extricate the feature of the image. Owing to the lack of medical labeling images for the training purpose, the unsupervised learning methods are incorporated [15].

## 3. Proposed CANN Model

The spot segregated from the original computed tomography image is given as the input to the CANN for the feature learning and representation process. The labelled data are used for attenuating the parameters of the CANN. The spot separated from the normal image is denoted by *x* ∈ *X*, *X*∁*R*^*m*∗*d*∗*d*^ where *m* is the total number of the input channel and *d* × *d* is the size of the input image. The labeled data are denoted by *y* ∈ *Y*, *Y*∁*R*^*n*^ where *n* represents the number of output classification. The hypothesis function is denoted as *f* : *X*⟶*Y*. Thus, in the proposed model, the hypothesis function *f* comprises of the multiple layers, and they are not connected to *X* to *Y* directly [16]. The center layer constitutes the three-pooling layer, three-convolution layer, and fully connected layer. The structure of the CANN is depicted in Figure 3.

The training data comprises of the labelled data and the unlabeled data, *UD* = {*x*, *x* ∈ *X*} and *D* = {*x*, *y*; *x* ∈ *X*, *y* ∈ *Y*} where *UD* denotes the unsupervised learning and the *D* represents supervised learning.

### 3.1. Standard Autoencoder

Thus, to perform data-driven representation learning, the supervised approach is initiated. The weights are applied to both the forward and the backward algorithms. The unlabeled input data are obtained from the unsupervised approach compared to that of the supervised approach. Autoencrypted method is applied in this study [18]. Later on, in performing several iterations, the cost function is validated. The input data is denoted by *I*; it corresponds to *m* dimension vector *I* ∈ *R*^*m*.

### 3.2. Convolution Autoencoder

Convolution autoencoder integrates convolution relation with the autoencrypted process. The values obtained from the output are patched via reverse convolution encrypted process. With the help of unsupervised training, the decoding and encoding performances are evaluated. The convolution encoder is represented by *f* (.), and the convolution decoder is denoted by *f* (..). Thus, the convolution autoencoder process includes *m* convolution kernels. *n* is considered as the number of input channel. The convolution kernel size is *d* × *d*.

The indiscriminate activation function is denoted by *σ*. This comprises of the various functions such as the elliptical function, inflated tangent function, and the rectified linear function (Relu).

(1) $$\begin{array}{c} \text{Relu}\left(x\right)=\left\{\begin{array}{c} x\;x\geq 0,\\ 0\;x<0. \end{array}\right. \end{array}$$

### 3.3. Pooling

The proposed CANN method is analogous to that of CNN. The pooling layer is connected to that of the convolutional layer. In the proposed CANN method, there exists the max pooling layer succeeding the convolutional layer [18].

(2) $$\begin{array}{c} o_{j}^{i}=\max\left(x_{j}^{i}\right). \end{array}$$

As per the size of the pooling layer, the input feature map is subdivided into *n* overlapping regions. Thus, *x*_*j*_^*i*^ denotes the region in the *i*th place and the feature map of the *j*th position, and the *o*_*j*_^*i*^ denotes the region in the *i*th place and the feature map of the *j*th position. In the pooling layer, the number of inputs is equal to that of the number of the output. After the pooling operation, the neurons in the feature map gets reduced. Thus, there is reduction in the computational complexity.

### 3.4. Cost Function

SoftMax layer is useful for categorizing according to the feature such as the max pooling layer, fully connected layer, and multiple convolution autoencrypted process. The bronchi computed tomography image is distinguished into several categories [19]. Basically, $\hat{y_{i}}$ denotes the random probability of the lumps and the absence of the lumps.

(3) $$\begin{array}{c} \hat{y_{i}}=\frac{e^{\left(o_{i}\right)}}{\sum_{k=1}^{2}e^{o_{k}}},i=0,1. \end{array}$$

The cost function is represented by *L*. In order to reduce *L*, the SGD is initialized. Thus, *y* is denoted as the sample data. The absence of lumps is represented by 1.

(4) $$\begin{array}{c} L=-\left(y\log\hat{y_{0}}+\left(1-y\right)\log\hat{y_{1}}\right). \end{array}$$

### 3.5. Training Parameters

#### 3.5.1. Convolution Autoencoder

The unsampled images are used for training the autoencrypted process. With the use of cost function, the gradient is calculated. Each sample is incorporated in the particular set of process; for each iteration, 50 samples are utilized; thus, the total number of samples per layer is denoted by 50 × (*N*/100). Hence, numerous channels are accompanied in the convolution encoder and decoder.

#### 3.5.2. Fully Connected Layer

The fully connected layer attains its input from the last layer called the polling layer. They are represented by 500 neurons. They are interconnected by the SoftMax classifier. At the fully connected layer, the parameter obtained via supervised learning is classified by the SoftMax classifier. For the categorizing process, 1800 labelled data are utilized [20].

#### 3.5.3. Algorithm of Training CANN

The training in CANN depends on both the supervised and unsupervised learning.

## 4. Results and Discussions

### 4.1. Dataset

The data used for classification are gathered in the health center present in China [18]. It comprises of the 5000 subjects' bronchi images from 2012 to 2015. Hence, for each lump, the clinician examines the region of interest portion. The data are segregated into several datasets, namely, D1, D2, and D3, respectively [21, 22].

D1: it constitutes 50000 samples from the unlabeled data of the unsupervised learning with the spot traced about of 64 × 64. These minute spots are examined in each subject [23]

D2: D2 comprises of the labelled data with the spot of 64 × 64, approximately of 3700 traces. These are determined by the clinician out of which 1890 constitutes diseased image and the 1810 comprises of normal images [24]

D3: the D3 comprises of the 500 pair of the labelled spot. These images are notified by the clinician. The resemblance predicted is from 1 to 4 where 4 is the greatest resemblance obtained and 1 is the lowest resemblance occurred. Thus, the 60 samples are vomited with the same resemblance of the value 2. It is determined that the midway resemblance value is vomited

### 4.2. Architecture Built with Convolution

In our study, two kinds of CANN are suggested; one is C-CANN and the other is S-CANN. The C-CANN is used for classification purpose, and the S-CANN is used for computing the similarity in the process [25]. The C-CANN comprises of three groups connecting the pooling and the convolution layer accompanied by the fully connected layer and a classifier. The specification is represented below. The experimentation is being carried out using MATLAB version 2018.

The input constitutes 64 × 64 spots.

There are three convolution layer and three max pooling layers.

C1: in the initial phase, the convolution layer comprises of 5 × 5  spots, and the total number of the convolutional part is 50

P1: the pooling area constitutes the size of about 2 × 2

C2: in the next phase, the convolution layer comprises of 3 × 3  spots, and the total number of the convolutional part is 50

P2: the pooling area constitutes the size of about 2 × 2

C3: the convolution layer comprises of 3 × 3  spots, and the total number of the convolutional part is 50

P3: the pooling area constitutes the size of about 2 × 2

S-CANN comprises of 8 layers similar to that of the C-CANN. The feature extraction is done for the set of images and the evaluation is carried out.

### 4.3. Classification

#### 4.3.1. Impact of Sample Images

Depending on the accuracy of the CANN and MCNN, the performance of them is computed. Thus, with the value of 2950 for both, the method execution is well performed. When it reaches 700 or 800, CANN produces better results [17].

#### 4.3.2. Performance Comparison and Classification

Both the CNN and the conventional learning method produce identical result in determining the spot in the bronchi; they both use the labelled dataset for classification. Utilizing the forward and backward propagation, the network parameters are learnt. MCNN is an alternative of the CNN. The performances of the CNN, CANN, and MCCNN are compared and the ROC is plotted. The performance metrics such as precision, recall, accuracy, and *F*1 score have been calculated as follows:

(5) $$\begin{array}{c} \text{Precision}=\frac{\text{TP}}{\text{TP}+\text{FP}}=\frac{\text{Total number of perfectly predicted true instances}}{\text{Total number of positive predictions as result of experimentation}}, \end{array}$$

(6) $$\begin{array}{c} \text{Accuracy}=\frac{\text{TP}+\text{TN}}{\text{TP}+\text{TN}+\text{FP}+\text{FN}}=\frac{\text{Total correct predictions}}{\text{Total predictions}}, \end{array}$$

(7) $$\begin{array}{c} \text{Recall}=\frac{\text{TP}}{\text{TP}+\text{FN}}, \end{array}$$

(8) $$\begin{array}{c} F1\text{ score}=2*\frac{\text{Recall}*\text{Precision}}{\text{Recall}+\text{Precision}}. \end{array}$$

The architecture of the CANN is utilized by the CNN and MCCNN. Thus, the precision, recall, accuracy, and *F*1 are obtained as 93.45%, 92.42%, 92.16%, and 92.19%, respectively. Despite the above method, the AE produces the precision, recall, accuracy, and *F*1 of about 78.45%, 77.24%, 77.43%, and 77.35%, respectively. The evaluation index of the CNN is 90.46%, 91.28%, 91.99%, and 91.56%. In addition to that, the evaluation index of MCNN is 91.22%, 90.65%, 89.14%, and 91.23%. Thus, the performance of the CANN is better compared to that of the CNN and MCCNN. Consequently, the AUC of AE, CANN, CNN, and MCCNN are 0.82, 0.98, 0.93, and 0.96, respectively, as shown in Figure 4.

### 4.4. Similarity Check

This technique enables clinician to predict the occurrence of the similar image. The similarity determination includes several parameters to be encountered; they are patterning, size, depth, boundary, etc.

Figure 5 shows the CANN performance regarding the similarity, classification, recall, accuracy, and *F*1. Thus, better results are obtained with the CANN method.  Figure 6 depicts the ROC over classification performance. It is inferred that the attained error rate is being realized with the value of 0.92 which is as close to unity.

## 5. Conclusion

In this study, the image analysis pair of approaches has been initialized. The traditional approach is time-consuming and it requires huge labor; thus, data-driven approach is capable of losing the data about the spot occurred in the bronchi, whereby due to scarcity of the labelled data, these two methods are not implemented. Hence, our study proposed a CANN-based data-driven model with the addition of numerous unlabeled data and the fewer labelled data are used. The main novelty which has been incorporated is the processing of data being made in a pattern of grid with minimal complexity and minimal noises, and it follows the adaptive strategy in acquiring the hierarchical feature subsets from minimal to maximal level patterns. This study evaluates the spot in the bronchi and performs classification task as well as the similarity validation is also performed. Through lot of experiments, the proposed method is estimated as best for classifying the spot in the bronchi. Our future work involves combining the data-driven feature learning with the base knowledge, and further process is performed.

## Figures and Tables

**Figure 1:** Illustration of the system defining the lack of unlabeled feature samples.

**Figure 2:** Illustration of CANN for medical image analysis.

**Figure 3:** Illustration over the structure of CANN for clinical image analysis [17].

**Figure 4:** The resultant characteristics of training sample count read over the accuracy of classification over MCNN and CANN.

**Figure 5:** Performance realization over the similarity of images.

**Figure 6:** Receiver operating characteristics over classification.

**Table 1:** Performance realizations over the various classifications.

Methodology	Precision (%)	Recall (%)	Accuracy (%)	AUC	*F*1 (%)
AE	78.45	77.24	77.43	0.82	77.35
CANN	93.45	92.42	92.16	0.98	92.19
CNN	90.46	91.28	91.99	0.93	91.56
MCCNN	91.22	90.65	89.14	0.96	91.23

## Data Availability

The data used to support the findings of this study are included in the article. Should further data or information be required, these are available from the corresponding author upon request.
